# Susceptible-Infected-Removed Mathematical Model under Deep Learning in Hospital Infection Control of Novel Coronavirus Pneumonia

**DOI:** 10.1155/2021/1535046

**Published:** 2021-10-27

**Authors:** Ting Liu, Yanling Bai, Mingmei Du, Yueming Gao, Yunxi Liu

**Affiliations:** ^1^First Department of Health Care, The Second Medical Center and National Clinical Research Center for Geriatric Diseases, Chinese PLA General Hospital, Beijing 100853, China; ^2^Department of Disease Control and Prevention, The First Medical Center of Chinese PLA General Hospital, Beijing 100853, China; ^3^Department of Rehabilitation Medicine, The Second Medical Center and National Clinical Research Center for Geriatric Diseases, Chinese PLA General Hospital, Beijing 100853, China

## Abstract

**Objective:**

This research aimed to explore the application of a mathematical model based on deep learning in hospital infection control of novel coronavirus (COVID-19) pneumonia.

**Methods:**

First, the epidemic data of Beijing, China, were utilized to make a definite susceptible-infected-removed (SIR) model fitting to determine the estimated value of the COVID-19 removal intensity *β*, which was then used to do a determined SIR model and a stochastic SIR model fitting for the hospital. In addition, the reasonable *β* and *γ* estimates of the hospital were determined, and the spread of the epidemic in hospital was simulated, to discuss the impact of basal reproductive number changes, isolation, vaccination, and so forth on COVID-19.

**Results:**

There was a certain gap between the fitting of SIR to the remover and the actual data. The fitting of the number of infections was accurate. The growth rate of the number of infections decreased after measures, such as isolation, were taken. The effect of herd immunity was achieved after the overall immunity reached 70.9%.

**Conclusion:**

The SIR model based on deep learning and the stochastic SIR fitting model were accurate in judging the development trend of the epidemic, which can provide basis and reference for hospital epidemic infection control.

## 1. Introduction

Novel coronavirus (COVID-19) is one of the current coronaviruses that can infect humans. On December 1, 2019, the first suspected case of COVID-19 was admitted to Jinyintan Hospital in Wuhan. After that, major hospitals in Wuhan received similar unidentified pneumonia patients one after another. The Wuhan Municipal Health Commission started an epidemiological investigation on December 29. On January 8, 2020, experts from the National Health Commission of China announced that the pathogen was a novel coronavirus [1]. According to the report of the Wuhan Health Commission on January 16, 41 new patients were reported in Wuhan, and 19 new cases were reported on January 19. Zhong Nanshan, head of the national expert team, said on January 20 that the disease was “human-to-human infectious” and that 217 new cases had been reported in Wuhan that day. The first cases were reported in Tianjin, Jiangxi, Zhejiang, and Henan provinces on January 21, marking the start of a full-scale outbreak of COVID-19 in China. As of March 1, the total number of confirmed cases in China has reached 80,000. Meanwhile, other countries have also reported the emergence of novel coronavirus infections. At present, the epidemic in China has been basically brought under control through continuous efforts. However, the epidemic continues to spread in other countries and the international situation is still grim. Against the background of global economic integration, the prevention and control of the epidemic must not be slackened. Currently, research on the COVID-19 model is mostly focused on the whole region [2]. There have been very few studies on hospitals. However, as the main battlefield of antiepidemic, it is very necessary to study the law of epidemic transmission and its control transmission. Specifically, health care workers are more likely to come into contact with patients and get sick. When health care workers get sick, it is not only a major blow to the health care system, but it also increases the risk to the general population. This is extremely detrimental to the prevention and control of the epidemic [3].

The use of models to study infection began as early as the 18^th^ century. The concept of establishing a model to solve the spread of infectious diseases was first proposed by Bernoulli when he studied the smallpox virus. By the middle of the 20^th^ century, scientists began systematic research on it. In 1926, Kermack and Mckendrick proposed the classic susceptible-infected-removed (SIR) warehouse model [4]. Various subsequent models were proposed based on that. Later, as the research on infectious disease models continues to deepen, scientists have further subdivided and characterized different infectious diseases, such as SIR and SIES models. In recent years, infectious disease models have developed rapidly with the development of computing power and big data. Many scientists modeled various infectious diseases. For example, some scientists established an SIR model with H1N1 as the research object and conducted a simulation study on it. There were many similar examples [5]. A large amount of research data showed that the establishment of infectious disease research models can effectively predict the development trend of infectious diseases, which was extremely important for the treatment and control of infectious diseases. The establishment of infectious disease models has occupied an irreplaceable and important position in modern infectious disease research.

Therefore, a SIR and stochastic model was established based on the data of the whole area of Beijing. Then, the data of the hospital was used as the research data to carry out empirical analysis on the model. It was expected to provide a basis for epidemic control and subsequent similar events.

## 2. Research Methods

### 2.1. Determination of SIR Model

Based on a set of ordinary differential equations, the population was divided into three types: susceptible, infected, and evacuated to establish the SIR model. Susceptible persons were represented by *S*_*t*_, which meant the number of susceptible persons, and the susceptible persons were defined as healthy people who had not yet been infected with the disease. Infected people were expressed by *I*_*t*_, which meant the number of people infected at time *t*, which was defined as a group that had been infected and could transmit from person to person. The migrants were represented by *R*_*t*_, which meant the number of migrants at time *t*, which was defined as the people who had been isolated, passed away, or recovered from immunity. Assuming that an epidemic occurred in a closed environment, the effects of normal birth rate and death rate were excluded, while population dynamics were ignored, and the total population was counted as *N*. Then,

(1) $$\begin{array}{c} S_{t}+I_{t}+R_{t}=N. \end{array}$$

In a unit of time at time *t*, if the infection intensity was *β*, the number of new infections was *βS*_*t*_*l*_*t*_. At time *t*, the number of people who were evacuated due to death and recovery was proportional to the number of infections. If the intensity of removal was calculated as *r*, the number of people who were evacuated was *rI*_*t*_. The specific SIR model with different parameters is shown in Figure 1.

### 2.2. Stochastic SIR Model

For the stochastic SIR model, the stochastic process is as follows: for a given probability space (Ω, *℘*, *P*) and a given parameter set *T*, each parameter satisfies *t* ∈ *T*. Then, *X*_*T*_={*X*(*t*, *w*), *t* ∈ *T*} is the random variable defined in the probability space (Ω, *℘*, *P*), and the corresponding random process *X*_*T*_={*X*(*t*, *w*), *t* ∈ *T*} in the probability space (Ω, *℘*, *P*) is denoted as {*X*(*t*), *t* ∈ *T*} or *X*(*t*). The discrete state continuous-time Markov process is as follows: in a random process {*X*(*t*), *t* ∈ *T*}, if there are any integer *n* and space states *I*, 0 ≤ *t*_0_ < *t*_1_ < *t*_2_ < …<*t*_*n*+1_,  *t*_*k*_ ∈ *T*,  *k*=0,1,2,…, *n*+1, and their states meet the following conditions:

(2) $$\begin{array}{c} P\left\{X\left(t_{n+1}\right)\leq i_{n+1}|X\left(t_{n}\right)=i_{n},\ldots ,X\left(t_{0}\right)=i_{0}\right\}=P\left\{X\left(t_{n+1}\right)\leq i_{n+1}|X\left(t_{n}\right)=i_{n}\right\}. \end{array}$$

Then, the stochastic process {*X*(*t*), *t* ∈ *T*} is a discrete state continuous Markov process. Continuous-time Markov chain: for the random process {*X*(*t*), *t* ∈ *T*}, if there are any integers *n* and state space *I*, *I*,  0 ≤ *t*_0_ < *t*_1_ < *t*_2_ < …<*t*_*n*+1_,  *t*_*k*_ ∈ *T*,  *k*=0,1,2,…, *n*+1, and the state satisfies the following conditions:

(3) $$\begin{array}{c} P\left\{X\left(t_{n+1}\right)=i_{n+1}|X\left(t_{n}\right)=i_{n},\ldots ,X\left(t_{0}\right)=i_{0}\right\}=P\left\{X\left(t_{n+1}\right)=i_{n+1}|X\left(t_{n}\right)=i_{n}\right\}. \end{array}$$

Then, the stochastic process {*X*(*t*), *t* ∈ *T*} is called the continuous-time Markov process, also known as the process *Q*−. The transition probability function: let {*X*(*t*), *t* ∈ *T*} be a continuous countable Marko chain; then, for any *i*, the transition probability *j* ∈ *E* is as follows:

(4) $$\begin{array}{c} pij\left(s,t\right)=P\left\{X\left(t\right)=j|X\left(S\right)=i\right\},\;s\leq t;\;i,\;j\in E. \end{array}$$

The above Markov chain is called the time homogenous Markov chain, and its transition probability is only related to the time interval and has nothing to do with the time selection. Therefore, when only the time homogenous Markov chain was considered, the above formula can be rewritten as follows:

(5) $$\begin{array}{c} p_{\mathrm{ij}}\left(t-s\right)=P\left\{X\left(t\right)=j|X\left(s\right)=i\right\}\\ =P\left\{X\left(t-s\right)=j|X\left(0\right)=i\right\},\;s\leq t;\;i,\;j\in I. \end{array}$$

The transition probability matrix is defined as follows:

(6) $$\begin{array}{c} P\left(t\right)=\left(pij\left(t\right)\right)i,\;j\in l. \end{array}$$

Chapman–Kolmogorov equation: for any *s*,  *t* ≥ 0,  *i*,  *j* ∈ *I*, there is the following equation:

(7) $$\begin{array}{c} p_{ij}\left(s+t\right)=\sum_{k\in I}p_{ik}\left(s\right)p_{kj}\left(t\right). \end{array}$$

Its matrix form is as follows:

(8) $$\begin{array}{c} P\left(s+t\right)=P\left(s\right)P\left(t\right),\;\forall s,\;t\in \left[0,\infty \right). \end{array}$$

The transition rate matrix is defined as follows:

(9) $$\begin{array}{c} A=\left(\begin{array}{cccc} a_{00} & a_{01} & a_{02} & \ldots a_{0n}\\ a_{10} & a_{11} & a_{12} & \ldots a_{1n}\\ a_{20} & a_{21} & a_{22} & \cdots a_{2n}\\ \vdots & \vdots & \vdots & \ddots \vdots \\ a_{n0} & a_{n1} & a_{n2} & \cdots a_{nn} \end{array}\right),\\ a_{ij}=\underset{\Delta t⟶0^{+}}{\lim}\frac{p_{ij}\left(\Delta t\right)-p_{ij}\left(0\right)}{\Delta t}=\left\{\begin{array}{c} \lim_{\Delta t⟶0}\frac{p_{ij}\left(\Delta t\right)}{\Delta t},\;i\neq j\\ \lim_{\Delta t⟶0}+\frac{p_{ij}\left(\Delta t\right)}{\Delta t},\;i=j \end{array}\right\}. \end{array}$$

According to ∑_*j*=0_^*∞*^*p*_*ij*_(Δ*t*)=1, the following equation is acquired:

(10) $$\begin{array}{c} 1-p_{ij}\left(\Delta t\right)=\sum_{j=0,j\neq i}^{\infty }p_{ij}\left(\Delta t\right)=\sum_{j=0,j\neq i}^{\infty }\left[a_{ij}\Delta t+o\left(\Delta t\right)\right]. \end{array}$$

Further, equation (11) is acquired:

(11) $$\begin{array}{c} a_{ii}=\underset{\Delta t⟶0^{+}}{\lim}\frac{-\sum_{j=0,j\neq 1}^{\infty }\left[a_{ij}\Delta t+o\left(\Delta t\right)\right]}{\Delta t}\\ =-\sum_{j=0,j\neq i}^{\infty }a_{ij}. \end{array}$$

Then, the following equation is obtained:

(12) $$\begin{array}{c} \sum_{j=0}^{\infty }a_{ij}=a_{ii}+\sum_{j=0,j\neq i}^{\infty }a_{ij}=0. \end{array}$$

The pure generative process is defined as follows:

(13) $$\begin{array}{c} P\left\{X_{t+dt}=j|X_{t}=i\right\}=\left\{\begin{array}{cc} \eta_{i}dt+o\left(dt\right), & j=i-1,\\ 1-\eta_{i}dt+o\left(dt\right), & j=i,\\ o\left(dt\right), & \text{others.} \end{array}\right) \end{array}$$

The birth and death processes are shown as follows:

(14) $$\begin{array}{c} P\left\{Xt+dt=j|Xt=i\right\}=\left\{\begin{array}{cc} \varsigma idt+o\left(dt\right), & j=i+1,\\ \eta idt+o\left(dt\right), & i=i-1,\\ 1-\left(\varsigma i+\eta i\right)dt+o\left(dt\right), & j=i,\\ o\left(dt\right), & \text{others.} \end{array}\right) \end{array}$$

A susceptible person was likely to become infected with a probability of *βS*_*t*_*I*_*t*_*dt*. The probability that an infected person would recover or die and become a remover is *γI*_*t*_*dt*. The probability of the above two occurrences is 1 − (*βS*_*t*_+*γ*)*I*_*t*_*dt*. Therefore, the transition probability of a binary random process {*S*_*t*_, *I*_*t*_, *t* ≥ 0} is as follows:

(15) $$\begin{array}{c} P\left\{{\left(S,I\right)}_{t+dt}=\left(i,j\right)|{\left(S,I\right)}_{t}=\left(m,n\right)\right\}. \end{array}$$

*β* and *γ* are removal coefficients. Specific infectious disease random models and least square cases under different coefficients are shown in Figures 2 and 3.

### 2.3. Parameter Estimation

*Least square method*: assuming unknown parameters *θ*=(*β*, *γ*), then the number of infected persons is *I*={*I*_*i*_, 1 ≤ *i* ≤ *N*}, the simulated value of the number of infected persons is *Y*(*θ*)={*y*_*i*_(*θ*), 1 ≤ *i* ≤ *N*}, and the residual is *V*=*Y*(*θ*) − 1 and the sum of squares SSE(*θ*) of the residual is as follows:
  (16) $$\begin{array}{c} \text{SSE}\left(\theta \right)={\left\|V\right\|}^{2}\\ =\sum_{i=1}^{N}{\left[y_{i}\left(\theta \right)-I_{i}\right]}^{2},\\ \left\{\begin{array}{c} \frac{\partial \text{SSE}\left(\theta \right)}{\partial \beta }=2\sum_{i=1}^{N}\left[y_{i}\left(\theta \right)-I_{i}\right]\frac{\partial y_{i}\left(\theta \right)}{\partial \beta },\\ \frac{\partial \text{SSE}\left(\theta \right)}{\partial \beta }=2\sum_{i=1}^{N}\left[y_{i}\left(\theta \right)-I_{i}\right]\frac{\partial y_{i}\left(\theta \right)}{\partial \gamma }. \end{array}\right) \end{array}$$
*Weighted least square method*: the recent data was given a large weight, while the long-term data was given a smaller weight, *w*^*N*−*i*^, 0 < *w* < 1, so the sum of squares SSE(*θ*) of the residual is as follows:
  (17) $$\begin{array}{c} \text{SSE}\left(\theta \right)={\left\|V\right\|}^{2}=\sum_{i=1}^{N}w^{N-i}{\left[y_{i}\left(\theta \right)-I_{i}\right]}^{2}+\sum_{i=N+1}^{M}{\left[y_{i}\left(\theta \right)-I_{i}\right]}^{2}. \end{array}$$

### 2.4. Empirical Study on COVID-19 in Hospital

Firstly, the SIR model was used to fit the epidemic situation of the hospital. In the SIR model, the whole population was classified into susceptible persons (*S*_*t*_), infected persons (*I*_*t*_), and displaced persons (*R*_*t*_). New diagnoses in hospital every day are shown in Figure 4. The number of newly diagnosed patients in hospital on a daily basis was consistent with the basic trend (*I*_*t*_) in the SIR model, so the SIR model can be used for fitting.

The parameter estimation of the SIR model was determined. The number of communicators was taken as the number of confirmed cases on the day minus the number of deaths and ceases on the day, and the cumulative number of deaths and ceases *R*_*t*_ was obtained as follows:

 
*I*_*t*_ = number confirmed on a day − cumulative number of deaths and cures.
 
*R*_*t*_ = cumulative number of deaths and cures

The number of persons hospitalized with the virus per day and the cumulative number of deaths and discharges are the number of evacuees. Then, the differential equation of SIR model is determined as follows:

(18) $$\begin{array}{c} \left\{\begin{array}{c} \frac{\text{d}s_{t}}{\text{dt}}=-\beta S_{t}I_{t},\\ \frac{\text{d}I_{t}}{\text{dt}}=\beta S_{t}I_{t}-\gamma I_{t},\\ \frac{\text{d}R_{t}}{\text{dt}}=\gamma I_{t}. \end{array}\right) \end{array}$$

The initial value was *I*_0_=241, *R*_0_=5, and the parameters to be evaluated were *S*_0_, *β*, and *γ*. The least square method was used to estimate the unknown parameters. First, the following definition is made to estimate *γ*:

(19) $$\begin{array}{c} \gamma \left(t\right)=\frac{R\left(t\right)-R\left(t-1\right)}{I\left(t-1\right)}. \end{array}$$

Thus, an estimate of 0.071 for *γ* is obtained, representing a recovery time of approximately 14 days per patient. Then, the least square estimation of *S*_0_ and *β* is carried out by using the estimated value of the obtained *γ*. The parameter domain of unknown parameters is [1.6 × 10^−4^, 1.8 × 10^−4^]  × [1600,1800], and the minimum value SSE is found to obtain the 3D stereogram and contour map. The least square estimate of *S*_0_ and *β* is as follows:

(20) $$\begin{array}{c} \hat{\beta }=1.68\times 10^{-4}{\hat{S}}_{0}=1672. \end{array}$$

The sum of squares of the residuals is as follows:

(21) $$\begin{array}{c} \text{SSE}=1.277\times 10^{5}. \end{array}$$

Then, the obtained *S*_0_=1672 is used for the least square estimation of *β* and *γ*. The parameter domain of unknown parameters is [1.6 × 10^−4^, 1.8 × 10^−4^] × [0.068, 0.076], the minimum value SSE within the range is found, and the 3D stereogram and contour map are obtained. The least squares estimate is as follows:

(22) $$\begin{array}{c} \hat{\beta }=1.684\times 10^{-4},\\ \hat{\gamma }=0.072. \end{array}$$

The corresponding residual peace is as follows:

(23) $$\begin{array}{c} \text{SSE}=1.2633\times 10^{5}. \end{array}$$

Parameter estimation of stochastic SIR model was as follows. Simulation steps of the stochastic process are as follows: (i) when *t*=0, the initial value is set as (*S*_0_, *I*_0_), *β*, *γ*. (ii) Random numbers with exponential distribution parameter *βS*_*t*_*I*_*t*_+*γI*_*t*_ are generated. (iii) Random number *k* that obeys uniform distribution *U*(0,1) is generated. Let *p*=*βS*_*t*_/*βS*_*t*_+*γ*, if *r* ≤ *p*, then (*S*_*t*+*dt*_, *I*_*t*+*dt*_)=(*S*_*t*_−1, *I*_*t*_+1). If *r* > *p*, then (*S*_*t*+*dt*_, *I*_*t*+*dt*_)=(*S*_*t*_, *I*_*t*_ − 1). (iv) The pretransfer state (*S*_*t*_, *I*_*t*_) is replaced with the posttransfer state (*S*_*t*+*dt*_, *I*_*t*+*dt*_); the previous process is repeated, and the process is terminated when *S*_*t*_=0 or when *I*_*t*_=0. The initial value is the same as that of the determined SIR model. The 25 × 25 grid is taken and the parameter domain is set as [2.5 × 10^−6^, 2.7 × 10^−6^] × [0.06, 0.08]. The minimum value of SSE is obtained via MATLAB, to draw the 3D stereogram and contour diagram. The least square estimate of the position parameter is as follows:

(24) $$\begin{array}{c} \hat{\beta }=2.588\times 10^{-6},\\ \hat{\gamma }=0.073. \end{array}$$

For the determined SIR model, the parameter fitting is substituted to extract the *I* change image. For the stochastic SIR model, the *I1* change image is also obtained by fitting its 10,000 orbits and averaging the values of the orbits on the whole point (Figure 5).

Although there is a certain gap in the image, considering the error that may occur in the operation is acceptable, the previous view is confirmed. The determined SIR model is regarded as the value of the whole point of the stochastic SIR model. When the stochastic SIR model has enough orbits to eliminate its random interference, the average value of the two is converged. The results of the two are similar, but the process is opposite. The determined SIR model is regarded as a macroscopic change. The stochastic SIR model is a microscopic action, which determines the change of a single person each time, which is more in line with objective changes. The changes in the three types of populations in the SIR model are not achieved overnight, so the stochastic SIR model is more convincing and more reasonable than the determined SIR model.

### 2.5. Statistical Methods

SPSS 22.0 data analysis software was used to analyze the data. The counting data were expressed as a percentage, and the measurement data were expressed as mean ± standard deviation. Analysis of variance was used to compare the data between groups, and *P* < 0.05 was considered statistically significant.

## 3. Results

### 3.1. Results Comparisons

The percentage error between the daily number of infected people and the actual number after February 12, the comparison between the fitting number of infected people and the real number, and the comparison of the number of displaced people are shown in Figure 6. For accurate data, the error control was better. There was not much difference between the fit number and the real number of infected people. There was a certain error in the fitting of the number of patients removed, which may be caused by a large number of patients during the epidemic and the failure of timely treatment and death of some patients or their self-healing.

### 3.2. Estimation of the Basic Regeneration Number

The variation of effective regenerative number and the relationship between basal regenerative number and herd immunity are shown in Figure 7. The effective number of regenerations in the first day was the basic number of regenerations, and the effective number of regenerations decreased as the susceptible person became infected. After the isolation of infected people and other measures, the susceptible group continued to shrink. The effect of herd immunity was achieved when the immune population reached 70.9% in the population, that is, when the basic regeneration number was less than or equal to 1. When the base regeneration number was less than or equal to 1, the outbreak would only occur in a small area and ended quickly.

### 3.3. Influences of Infection Intensity on the Development of the Epidemic

The number of people infected under different infection intensities is shown in Figure 8. When *β* decreased to 30%, the peak number of infections decreased significantly, and when *β* decreased to 50%, the peak number of infections decreased further. As *β* went down, the ability of the new coronet to infect went down, so did the peak number of infections. Although it had a small effect on the total number of people infected, it can slow the progression of the epidemic and reduce the pressure on medical care by delaying the peak.

### 3.4. The Impact of Vaccines and Other Measures on the Outbreak

Figures 9 and 10 show the comparison of 30% vaccine-covered and 30% vaccine-covered and quarantined with no measures of infection. When vaccine coverage reached 30 percent, both the peak daily patient count and the cumulative number of patients declined by 34 percent. When the vaccine was covered by 30% and the isolation measures were taken, the peak daily cumulative number of patients and the total cumulative number of patients decreased further, by 70%. Vaccine coverage and isolation control were proven effective.

## 4. Discussion

Infectious diseases have always been one of the common and dangerous factors threatening human life and health. Because of their tendency to spread on a large scale, they lead to not only the demise of individuals but also the demise of species, nations, and even civilizations. Civilizations have been wiped out by infectious diseases throughout human history. Early Spanish explorers to Latin America, for example, discovered that the Mayas and Incas who had lived there for generations were wiped out by smallpox [6]. In addition to that, there have been a number of similar epidemics in human history, such as the plague in the heartland of Mongolia in the east and the Black Death in the west. These have caused great disasters to human society. There were many similar cases. In ancient China, there were 261 plague cases recorded, and some scholars even found records of plague in oracle bones. To sum up, infectious diseases have a huge impact on human society [7]. Human beings have never stopped fighting against infectious diseases. As early as the pre-Qin period, China cut off the source of infection through isolation and other means. Modern western scholars performed smallpox virus research, and the smallpox virus has been eliminated. Another example is the outbreak of plague in Northeast China during the period of the Republic of China. Liande Wu, a medical doctor, was ordered to stop a deadly infectious disease [8].

With the continuous development of modern science and technology and medical treatment, the medical level has improved a lot. Human research on infectious diseases is deepening, but bacteria and viruses are also constantly mutating and evolving. All kinds of new pathogens emerge in an endless stream. For example, there was the outbreak of hepatitis C in China in 1989 and the middle east respiratory syndrome (MERS), which was prevalent in a small area in the Middle East a few years ago, and SARS which was prevalent in a large area in the world in 2003. In recent years, as the range of human activities continues to expand, the boundary between human beings and nature is getting lower and lower, which leads to the increasing probability of human being being infected with infectious diseases [9]. For example, the H1NI virus which emerged in 2009 originally appeared in birds. After continuous mutation, it eventually became parasitic on people. It took the lives of tens of thousands of people in the United States and caused a huge burden to the American society. There are more than 3,000 known viruses, and this is just the tip of the iceberg. Human beings have a long way to go in the prevention and treatment of infectious diseases [10].

Using models to study infection began as early as the 18^th^ century. The concept of establishing a model to solve the spread of infectious diseases was first proposed by Bernoulli when he studied the smallpox virus. By the middle of the 20^th^ century, scientists began systematic research on it. In 1926, Kermack and Mckendrick proposed the classic susceptible-infected-removed (SIR) warehouse model [11]. Various subsequent models were proposed based on that. Later, as the research on infectious disease models continues to deepen, scientists have further subdivided and characterized different infectious diseases, such as SIR and SIES models. In recent years, infectious disease models have developed rapidly with the development of computing power and big data. Many scientists modeled various infectious diseases [12]. For example, some scientists established an SIR model with H1N1 as the research object and conducted a simulation study on it [13]. There were many similar examples. A large amount of research data showed that the establishment of infectious disease research models can effectively predict the development trend of infectious diseases, which was extremely important for the treatment and control of infectious diseases. The establishment of infectious disease models has occupied an irreplaceable and important position in modern infectious disease research. Therefore, the SIR model and SIR stochastic model based on deep learning were established in this work to explore the development law of the COVID-19.

COVID-19 is one of the current coronaviruses that can infect humans. On December 1, 2019, the first suspected case of COVID-19 was admitted to Jinyintan Hospital in Wuhan. After that, major hospitals in Wuhan received similar unidentified pneumonia patients one after another. The Wuhan Municipal Health Commission started an epidemiological investigation on December 29. On January 8, 2020, experts from the National Health Commission of China announced that the pathogen was a novel coronavirus. According to the report of the Wuhan Health Commission on January 16, 41 new patients were reported in Wuhan, and 19 new cases were reported on January 19. Zhong Nanshan, head of the national expert team, said on January 20 that the disease was “human-to-human infectious” and that 217 new cases had been reported in Wuhan that day [14]. The first cases were reported in Tianjin, Jiangxi, Zhejiang, and Henan provinces on January 21, marking the start of a full-scale outbreak of COVID-19 in China. As of March 1, the total number of confirmed cases in China has reached 80,000. Meanwhile, other countries have also reported the emergence of novel coronavirus infection. At present, the epidemic in China has been basically brought under control through continuous efforts. However, the epidemic continues to spread in other countries and the international situation is still grim. Against the background of global economic integration, the prevention and control of the epidemic must not be slackened. Currently, research on the COVID-19 model is mostly focused on the whole region. There have been very few studies on hospitals. However, as the main battlefield of antiepidemic, it is very necessary to study the law of epidemic transmission and its control transmission. Specifically, health care workers are more likely to come into contact with patients and get sick. When health care workers get sick, it not only is a major blow to the health care system but also increases the risk to the general population this is extremely detrimental to the prevention and control of the epidemic [15].

Therefore, a retrospective analysis of the occurrence of COVID-19 in hospital was performed by using the SIR model based on deep learning and the SIR stochastic model. Based on the SIR model, the COVID-19 epidemic situation in Wuhan was studied, and the research time was from January 23, 2020, to March 31, 2020. The law of the spread of the epidemic was discovered through daily epidemic information and restoring of its development process. Finally, some valuable information was obtained through the model, which had positive significance for potential prevention and control work in the future. The determined SIR model and stochastic SIR model were taken as the core, and then the Wuhan area was modeled. First, *S*_0_ was used as the parameter to be estimated, and its range was determined by MATLAB to find a better fitting effect. Then, the obtained o value was used to find *β* and *Y* suitable for the Wuhan area. In the stochastic SIR model, the continuous-time Markov Chain was used to fit *S*_0_, *B*, and *y* again. The residual square SSE chart of the daily number of infected persons was plotted through the computer running 5,000 orbits, and the extreme points of the infection intensity *B* and the recovery intensity were found, which were compared with the determination of the SIR equation, and the error was within a reasonable range. Then, a simulation of 10,000 orbits was implemented to draw a simulation diagram of the three groups of people, which showed that the determined SIR model was the mean process of the stochastic SIR model without considering the covariance. Finally, the different results of changing the intensity of infection and the intensity of removal on the development of the epidemic were discussed. It was found that quarantine, vaccine, and other measures had an impact on the development of the epidemic. The intensity of infection was a key factor affecting the outbreak. It was also found that the SIR model and stochastic model based on deep learning had an ideal prediction effect on the development trend of the epidemic.

## 5. Conclusion

The deep learning SIR model and stochastic SIR model were used to retrospectively study the occurrence of COVID-19 in hospital. It was found that the above two models were accurate in predicting the development trend of the epidemic and had a high prospect in hospital epidemic control. In addition, vaccine, isolation, and infection intensity had a great impact on the development of the epidemic, and the epidemic can be controlled from these three aspects when similar situations occur in the future. However, due to the limited sample and space, the study on this issue is not comprehensive and in-depth enough. In future study and work, it will expand the sample for further study.

This work was developed based on the determined SIR model and stochastic SIR model. Although some effects were achieved in predictive analysis, there are many shortcomings. First, the variability of *B* and *y* is not fully considered, which are set as a constant. From the beginning to the end of the epidemic, *B* and *y* may change due to various reasons such as the government's control and the update of medical resources, so the patient's ability to get infected should go down, and the level of recovery should go up as various drugs are tested, In the future, we can consider its time-varying function to conform to objective facts. Secondly, the description index of the model is too single. For the most critical infection intensity and recovery intensity, population mobility, medical resource level, and aging rate in each region are different, which are all important parameters affecting the accuracy of the model. In the future, it can be considered as a breakthrough to continuously optimize model equations and parameters to achieve more accurate results.

## Figures and Tables

**Figure 1:** SIR epidemic model with different parameters.

**Figure 2:** Random SIR epidemic model under different parameters.

**Figure 3:** Least square case.

**Figure 4:** New diagnoses and statistics in hospital every day. (a) Newly diagnosed infections per day. (b) The number of new infections per day.

**Figure 5:** Fitting graph of the number of daily infected persons of determined SIR model and stochastic SIR model.

**Figure 6:** Comparison of fitting results. (a) Percentage of error between the daily infected number and the actual number. (b) Comparison between the actual number of people and the fitted number. (c) Comparison of the number of migrants.

**Figure 7:** Analysis of basic regenerative number. (a) The variation of the base regeneration number. (b) Relationship between basal regenerative number and the proportion of herd immunity.

**Figure 8:** Number of infected persons under different infection intensities.

**Figure 9:** Comparison of the number of infected persons with vaccine coverage and those without vaccine coverage.

**Figure 10:** Comparison of 30% vaccine coverage plus isolation and no measures.

## Data Availability

The data used to support the findings of this study are available from the corresponding author upon request.

## References

[1] Wicker S. (2019). BK 3101 - i. *Internist*.

[2] Li H., Bai R., Zhao Z. (2018). Application of droplet digital PCR to detect the pathogens of infectious diseases. *Bioscience Reports*.

[3] Lounis M., Bagal D. K. (2020). Estimation of SIR model’s parameters of COVID-19 in Algeria. *Bulletin of the National Research Centre*.

[4] Lv Z., Li X., Li W. (2017). Virtual reality geographical interactive scene semantics research for immersive geography learning. *Neurocomputing*.

[5] Zhihan L., Xiaoming L., Weixi W., Baoyun Z., Jinxing H., Shengzhong F. (2018). Government affairs service platform for smart city. *Future Generation Computer Systems: FGCS*.

[6] Cooper I., Mondal A., Antonopoulos C. G. (2020). A SIR model assumption for the spread of COVID-19 in different communities. *Chaos, Solitons & Fractals*.

[7] Ball F., Britton T., Leung K. Y., Sirl D. (2019). A stochastic SIR network epidemic model with preventive dropping of edges. *Journal of Mathematical Biology*.

[8] Chladná Z., Kopfová J., Rachinskii D., Rouf S. C. (2020). Global dynamics of SIR model with switched transmission rate. *Journal of Mathematical Biology*.

[9] Libertucci J., Young V. B. (2019). The role of the microbiota in infectious diseases. *Nature Microbiology*.

[10] Kak G., Raza M., Tiwari B. K. (2018). Interferon-gamma (IFN-*γ*): e. *Biomolecular Concepts*.

[11] Prodanov D. (2020). Analytical parameter estimation of the SIR epidemic model. Applications to the COVID-19 pandemic. *Entropy*.

[12] Comunian A., Gaburro R., Giudici M. (2020). Inversion of a SIR-based model: a critical analysis about the application to COVID-19 epidemic. *Physica D: Nonlinear Phenomena*.

[13] Chung J. Y., Thone M. N., Kwon Y. J. (2021). COVID-19 vaccines: the status and perspectives in delivery points of view. *Advanced Drug Delivery Reviews*.

[14] Han H. J., Nwagwu C., Anyim O., Ekweremadu C., Kim S. (2021). COVID-19 and cancer: from basic mechanisms to vaccine development using nanotechnology. *International Immunopharmacology*.

[15] Taleghani N., Taghipour F. (2021). Diagnosis of COVID-19 for controlling the pandemic: a review of the state-of-the-art. *Biosensors and Bioelectronics*.

